The article "The Efficacy of Exposure and Response Prevention for Geriatric Obsessive Compulsive Disorder: A Clinical Case Illustration" was published in 2012. Journal: Case Rep Psychiatry.

# The Efficacy of Exposure and Response Prevention for Geriatric Obsessive Compulsive Disorder: A Clinical Case Illustration

**DOI:** 10.1155/2012/394603

**Published:** 2012-12-17

**Authors:** Mairwen K. Jones, Bethany M. Wootton, Lisa D. Vaccaro

**Affiliations:** ^1^The University of Sydney Anxiety Disorders Clinic, Discipline of Behavioural and Social Sciences in Health, Faculty of Health Sciences, The University of Sydney, Cumberland Campus, East Street, Lidcombe, NSW 2141, Australia; ^2^Centre for Emotional Health, Department of Psychology, Macquarie University and Discipline of Behavioural and Social Sciences in Health, The Faculty of Health Sciences, The University of Sydney, Lidconbe, NSW 2113, Australia; ^3^Discipline of Behavioural and Social Sciences in Health, Faculty of Health Sciences, The University of Sydney, Cumberland Campus, East Street, Lidcombe, NSW 2141, Australia

## Abstract

Obsessive compulsive disorder (OCD) is one of the most frequently occurring psychiatric conditions in older adults. While exposure and response prevention (ERP) is considered the most effective psychological treatment for children and adults with OCD, research investigating its effectiveness for older adults is scarce. This clinical case study investigates the effectiveness of ERP in an 80-year-old man with a 65-year history of OCD. The client received 14 individual, 50-minute ERP treatment sessions. Clinician-based Y-BOCS scores reduced by 65% from 20 (moderate) at pretreatment to 7 (subclinical) at 7-month posttreatment followup. OCI-R total scores reduced by 45% from 38 at baseline to 21 at 7-month follow-up. Despite his long history of the disorder, ERP was effective and well tolerated. The application of ERP for older adults with OCD, including age-specific modifications that may be required for this treatment approach, is discussed.

## 1. Introduction

Obsessive compulsive disorder (OCD) is an anxiety disorder characterised by intrusive obsessions and/or repetitive, time-consuming compulsions [1]. It is a particularly disabling condition with significant impairment in functioning [2] and a high burden of disease and injury [3]. OCD is a common condition with twelve month prevalence estimates in adults noted to range from 0.6% to 1.9% [4]. The development of OCD after the age of 50 years is considered to be rare and is often associated with structural cerebral damage [5]. However, a considerable number of older adults are likely to be living with OCD [6], since they may have had the condition for many years and either not sought treatment or received inappropriate or ineffective treatments in the past [4]. For example, Grenier et al. [7] classified 1.5% of a sample of 2798 community dwelling adults aged over 65 years as probable OCD cases. Additionally, significant numbers of elderly people with OCD are seen in clinical practice [8]. In one sample of 183 patients seeking treatment for OCD 12% were older than 50 years [9]. As such, it has been argued that OCD is likely to be one of the most frequently occurring psychiatric conditions in this age group [10]. 

The article "The Efficacy of Exposure and Response Prevention for Geriatric Obsessive Compulsive Disorder: A Clinical Case Illustration" was published in 2012. Journal: Case Rep Psychiatry.

Additionally, older adults with untreated OCD are likely to experience significant disability across multiple areas of functioning [7], which could limit their ability to live independently in the community and substantially decrease their quality of life. Living with longstanding, persistent anxiety can also have a negative impact on the older adult's physical health, by compromising the cardiovascular system and increasing the individual's risk of coronary heart disease [11]. Therefore, research that can advance our understanding of which treatments are most efficacious for the older adult with OCD is clearly warranted. It is perhaps surprising, therefore, that a significant lack of research in this area has been identified [6, 10, 12, 13]. 

Exposure and response prevention (ERP) is considered one of the most effective treatments for OCD [14]. ERP is a psychological treatment that involves developing a hierarchy of feared situations which the client gradually confronts until habituation occurs [15]. Treatment usually commences with items from the hierarchy that are moderately difficult, after which the client confronts more difficult situations. While the client is expected to experience anxiety and discomfort when confronting the different items on the hierarchy [15], this approach isn't associated with the physical side effects that typically occur with many of the pharmacological agents used to treat OCD. As noted by Carmin et al. [16] the use of pharmacotherapy can be particularly problematic for the elderly OCD client, and their use needs to be carefully considered. 

The success of cognitive and behavioural treatments that include ERP has been demonstrated across numerous studies in both adult [17] and pediatric [18] OCD populations. However, individuals over the age of 65 years have generally been excluded from these treatment trials [19–21]. As such, the generalisability of these methods to elderly populations remains largely undocumented [22]. Instead, the management of anxiety in this population is likely to be extrapolated from research employing younger age group, or based on personal clinical experience [23]. 

A limited amount of research exploring treatment efficacy for geriatric OCD has been conducted, but it is at a relatively early stage. For example, recent research demonstrated the effectiveness of the cognitive intervention Danger Ideation Reduction Therapy for an 86-year-old man who had lived with OCD for more than six decades [24]. Several researchers have also demonstrated in single case studies the efficacy of ERP when combined with other OCD treatment approaches. These have included ERP with pharmacotherapy for older adults who developed late onset OCD following a basal ganglia infarct [22], or following stressful life events [25]. Hirsch et al. [26] demonstrated the effectiveness of a combined approach that included both ERP and cognitive interventions for an 80-year old man who had experienced OCD for 50 years. While research investigating the efficacy of ERP as a standalone intervention for the elderly OCD client is lacking, some reports have appeared in the literature. 

The article "The Efficacy of Exposure and Response Prevention for Geriatric Obsessive Compulsive Disorder: A Clinical Case Illustration" was published in 2012. Journal: Case Rep Psychiatry.

Two case reports examining the benefits of ERP for older adults with OCD were presented by Calamari and Cassiday [10]. The first case involved a 77-year-old female living with OCD hoarding. Some age-specific modifications to the ERP treatment were required which included the use of diaphragmatic breathing and relaxation skills to assist with managing the severe anxiety and feared bodily sensations during some exposure sessions. This treatment approach was found to be beneficial [10]. The second case involved an 86-year-old female with severe OCD symptoms that she had experienced since the age of five years. These included scrupulosity, doubting, and excessive hand washing. Since her physician was concerned about the possible negative impact on the client's blood pressure due to elevated anxiety resulting from the ERP protocol, single sessions were conducted weekly over eight weeks, instead of multiple sessions each week. While the client continued to have pronounced OCD symptoms she reported she was happy with the reduction in her OCD symptoms. It is worth noting that both clients had reported multiple hospitalisations and prior ineffective treatments.

Carmin and Wiegartz [13] also describe two cases of older adults with severe OCD who received ERP treatment. The first patient was a 78-year-old male with a recent onset of OCD whose rituals occupied him for up to eight hours a day. ERP treatment was modified due to the existence of physical health problems including hypertension and basal ganglia infarcts. ERP was not commenced until his hypertension was medically controlled, and he was taught progressive muscle relaxation training and diaphragmatic breathing as anxiety management strategies to help minimise blood pressure elevation. Additionally, simplification and repetition of psycho-educational interventions were carried out to facilitate understanding and retention, since the patient had difficulties with abstraction, possibly due to the basal ganglia infarcts. The second patient was a 74-year-old male with a 60-year history of the condition. He had previously required hospitalisation for his OCD and been prescribed both medications and ECT but had never undertaken ERP. 

The article "The Efficacy of Exposure and Response Prevention for Geriatric Obsessive Compulsive Disorder: A Clinical Case Illustration" was published in 2012. Journal: Case Rep Psychiatry.

Both patients commenced individual ERP sessions twice daily for 60 to 90 minutes. The first patient's score on the Yale Brown Obsessive Compulsive Disorder Scale (Y-BOCS) [27, 28] reduced from 24 at pretreatment to 19 on the day of discharge (day 21), and at 12 weeks posttreatment the Y-BOCS was 2. These treatment gains were maintained for at least one year. The second patient's Y-BOCS was 40 at pretreatment and 16 on the day he was discharged (day 23). However, while no follow-up Y-BOCS score was reported, the researchers noted that soon after returning home he had commenced ritualising to pretreatment levels. This patient had a long standing history of OCD, unlike the first patient who had experienced OCD for less than a year and experienced significant symptom reduction that was maintained over time. Carmin and Wiegartz [13] suggest that duration of symptoms may have been responsible for these different treatment outcomes. 

Another single case study examining the effectiveness of ERP was carried out by Colvin and Boddington [29] with a 78-year old woman who developed OCD symptoms after her house was flooded. ERP was conducted in the client's home over an eight-hour period and was shown to be effective. Yale Brown Obsessive Compulsive Disorder Scale (Y-BOCS) [27, 28] scores reduced from 35 at pretreatment to 12 at posttreatment and 11 at two-month followup. Further findings that provide support for the effectiveness of ERP for the elderly OCD patient were reported by Carmin et al. [16]. They found no significant differences in treatment response to ERP between two groups of clients matched for sex, depression, and OCD clinical severity. One group consisted of ten adults aged over 60 years, the other group employed ten young adults. The fact that both groups improved is particularly noteworthy since those in the older group had experienced OCD symptoms for a significantly greater period than the younger adults. 

In more recent research Price and Salsman [6] demonstrated that 20 sessions of ERP were effective for an 82-year-old male who had late-onset OCD with no identifiable neurobiological pathology. The dominant OCD symptoms included obsessions concerning contamination, being robbed or disturbed, and cleaning and checking compulsions. Some minor-age-relevant modifications were used including the placement of signs written in large font in his bathroom reminding him how long he should spend washing his hands and the selection of therapy rooms that were easily accessible and also had comfortable seating. Yale Brown Obsessive Compulsive Disorder Scale (Y-BOCS) [27, 28] scores reduced from 18 at pretreatment to 13 at posttreatment, and at 12-month followup Y-BOCS had reduced to zero. However, as the client had lived with OCD for less than a year before receiving treatment the researchers suggest that similar results may not be observed in older adults with longstanding OCD.

The article "The Efficacy of Exposure and Response Prevention for Geriatric Obsessive Compulsive Disorder: A Clinical Case Illustration" was published in 2012. Journal: Case Rep Psychiatry.

While research investigating response to ERP treatment in elderly clients with OCD is extremely scarce, the findings presented above demonstrate that this approach is very effective for some elderly people with OCD. However, some of the findings indicate that ERP may not be as beneficial for people who have experienced the condition for a long period of time. For example, Calamari and Cassiday [10] noted that their female client with severe OCD who had been living with the condition for approximately 80 years displayed some OCD symptom reduction but was left with pronounced OCD symptoms at the end of ERP treatment. Similarly, Carmin and Wiegartz [13] found that their 74-year-old male client who had lived with OCD for approximately 60 years experienced a decrease in symptoms from pretreatment to posttreatment, but commenced ritualising to pretreatment levels after returning home. 

We aim to augment the literature concerning the appropriateness of ERP for older adults by presenting a clinical case study that investigates the efficacy of ERP for an 80-year-old client. Further, given that the client has a 65-year-history of OCD we will be able to assess its effectiveness for someone with longstanding OCD. 

## 2. Materials and Methods

### 2.1. Participant

The participant who we will refer to as “Peter” was an 80-year-old married, retired man who reported a 65-year history of OCD. Peter presented to the University of Sydney Anxiety Disorders Clinic to take part in a 14-week randomised controlled trial investigating the efficacy of treatments for OCD. The participant gave informed consent, and the trial was authorised by the University of Sydney Ethics Committee. Peter presented with obsessions relating to fears of harming himself or others, which resulted in repeated checking of locks of his home, vehicle, and electrical appliances, asking his wife for reassurance, and asking his wife to complete his compulsions. Peter also had significant sexual and religious obsessions, which resulted in mental rituals of prayer and avoidance. 

In the past Peter had consulted a number of mental health professionals for treatment of his OCD. He had previously undertaken early psychological treatments including thought stopping and aversion therapy but had never received ERP. Peter had also been treated with pharmacological interventions, and at the time of the current treatment Peter was medicated on 50 mg of sertraline. He had been stable on this dose for four years and remained on this medication dosage throughout the treatment and follow-up periods of the current study, since changing the dose at this time would have meant we would not have been able to determine whether it was the ERP treatment or medication treatment that led to changes in OCD symptoms. Peter had previously abused alcohol from the age of 52 to 65, but for the past 15 years he had been abstinent from alcohol. At the time of treatment Peter did not have any other comorbid psychological problems. 

The article "The Efficacy of Exposure and Response Prevention for Geriatric Obsessive Compulsive Disorder: A Clinical Case Illustration" was published in 2012. Journal: Case Rep Psychiatry.

### 2.2. Treatment

Peter was randomly allocated to the ERP treatment condition. This intervention was based on the ERP package described by Andrews et al. [15] which is strictly behavioral and does not employ any cognitive interventions. The treatment involved developing a hierarchy of feared situations which were each gradually confronted until habituation occurred. Treatment commenced with items from the hierarchy that were moderately difficult for Peter and continued to the most difficult; that is, the situations he feared the most. Where possible, therapist-guided exposure was conducted in session; however, the majority of exposure tasks were conducted by the client at his home. The treatment was conducted by the second author, a registered clinical psychologist. Treatment consisted of 14, 50-minute weekly treatment sessions in total. 

### 2.3. Measures

Yale Brown Obsessive Compulsive Disorder Scale (Y-BOCS) [27, 28] was used. Consistent with other OCD treatment trials, the main outcome measure was the Y-BOCS. The Y-BOCS is a 10-item clinician administered questionnaire that assesses the nature and severity of OCD. Each question is scored on a 4-point Likert scale (0; no symptoms, 4; severe symptoms). Total scores range from 0–40, and higher scores reflect greater impairment. 

Obsessive Compulsive Inventory-Revised (OCI-R) (Foa et al.) [30] was also used. The OCI is an 18-item self-report questionnaire that assesses OCD symptoms across six subtypes (washing, checking, ordering, obsessing, hoarding, and mental neutralising). Each question is rated on a 5-point Likert scale. Scores on each subscale range from 0–12, and total scores range from 0–72, with higher scores indicating greater impairment. 

### 2.4. Data Analysis

All data was analysed with SPSS (version 18.0) (SPSS Inc., Chicago, IL, USA).

The article "The Efficacy of Exposure and Response Prevention for Geriatric Obsessive Compulsive Disorder: A Clinical Case Illustration" was published in 2012. Journal: Case Rep Psychiatry.

## 3. Results and Discussion

Y-BOCS data were collected at baseline and 7-month posttreatment. The scores on the Y-BOCS reduced 65% from 20 (moderate), to 7 (subclinical) at 7-months posttreatment. For the OCI-R total scores reduced by 45% from 38 at baseline to 21 at 7-month followup. Scores on all subscales were reduced after treatment. On the checking subscale, which was Peter's dominant compulsive behaviour, scores reduced 56%. At the end of treatment Peter stated that “If I had received treatment 60 years ago my life would have been so much better.” 

This clinical case study documents the successful treatment of an 80-year-old man with a 65-year history of OCD. The results add to existing evidence that ERP can be both an acceptable and effective treatment for older adults and are consistent with some findings reported by other researchers [6, 10, 13, 16, 29]. Additionally, the issue of whether older adults with OCD who have a long-standing history of the condition can benefit from ERP has been recently raised by researchers in this area [6], and some findings have provided support for this view [10, 13]. However, the findings presented in the current study provide evidence that ERP can be successful for an older adult with longstanding OCD. 

Some limitations of the current study need to be acknowledged. Despite Peter's long history of OCD, his OCD was of only moderate severity and not complicated by any psychological comorbid conditions. Additionally, he was not cognitively impaired and was relatively physically healthy. This may not be the case for all older adults with OCD, and these issues may pose complications in ERP treatment. Further, while age-related modifications to ERP therapy were not required for this client, they may be needed when working with other older adults with OCD and should therefore be considered on a case by case basis. For example, these may include the use of motivation enhancement for older clients who have been living with OCD for many years and experienced multiple ineffective treatments that have left them pessimistic or sceptical about treatment [10]. 

## 4. Conclusion

 While older adults with OCD have, to some extent, been neglected to date, we believe there is reason to be optimistic that older adults with OCD, like younger adults and children, can benefit from standard OCD treatments, such as ERP. Additionally, ERP may have specific benefits for the elderly OCD client over other OCD treatments such as pharmacological approaches that can be potentially harmful for elderly clients [16]. Only future research including further case investigations and controlled studies will confirm whether this optimism is warranted.
